The article "Nexus between energy efficiency, green investment, urbanization and environmental quality: Evidence from MENA region" was retracted in 2025. Reasons: unreliable results or conclusions; concerns about the article.

# Nexus between energy efficiency, green investment, urbanization and environmental quality: Evidence from MENA region

**DOI:** 10.1371/journal.pone.0295628

**Published:** 2023-12-29

**Authors:** Chen Gang, He Sha, Md Qamruzzaman

**Affiliations:** 1 School of Economics and Management, Southwest Petroleum University, Sichuan Province, China; 2 Xi’an Bomay Electric Industries Co., Ltd, Xi’an, China; 3 Southwest Petroleum University, Sichuan Province, China; 4 School of Business and Economics, United International University, Dhaka, Bangladesh; University of Pitesti, Romania; Institute of Doctoral and Post-doctoral Studies, University Lucian Blaga of Sibiu, ROMANIA

## Abstract

Environmental protection holds a paramount position in the pursuit of sustainable development. The existing body of literature has extensively examined various driving forces for environmental enhancement, including renewable energy sources, innovation, and governmental interventions. This study aims to assess the impact of green investment, energy efficiency, and urbanization on achieving environmental sustainability in the MENA region during the period 2004–2019. A comprehensive set of econometric tools has been employed to achieve this goal, including the CADF and CIPS panel unit root tests, error correction-based panel cointegration analysis, Cross-sectional ARDL, and asymmetric ARDL models. The key findings of this research are as follows: Cross-sectional dependency and homogeneity tests demonstrated that the research units shared common dynamics and heterogeneity properties. The stationarity tests based on CIPS and CADF indicated that all variables became stationary after the first differencing. The panel cointegration analysis established a long-term relationship between green investment (GI), energy efficiency (EE), urbanization (UR), and environmental sustainability (ES) in MENA nations. Empirical model estimations using Cross-sectional ARDL revealed significant contributions of GI, EE, and UR to ES in the long and short run. The asymmetry assessment uncovered a nonlinear relationship between the explanatory and dependent variables, both in the long and short run. Specifically, the asymmetric coefficients of GI, EE, and UR displayed negative statistical significance at the 1% level, highlighting their significant roles in promoting environmental sustainability. In light of these findings, this study provides valuable insights for policymakers to formulate strategies to further environmental sustainability in the MENA region.

## 1. Background of the study

In the 21st century, the world faces various difficulties, including growing urbanization, environmental deterioration, and climate change. Green investments in energy efficiency have arisen as a promising solution to such challenges [1–4]. The international community has recognized the significance of green finance in achieving sustainable development objectives and reducing carbon emissions. Urbanization is a significant source of economic growth and progress but also exerts substantial environmental stress. Cities account for a disproportionate percentage of greenhouse gas emissions and energy and resource usage. At the same time, more and more people are beginning to understand the value of sustainable development and the part that green investments and energy efficiency play in securing a sustainable future for the environment [5–12]. The finance of the transition to a low-carbon economy is also dependent on green investment. There is an increasing need for finance to fund essential infrastructure and technologies as more nations and cities commit to decreasing carbon emissions [13]. Some global implications of the connection among green investment, energy efficiency, urbanization, and environmental sustainability: Green investments can boost urban energy efficiency. As more and more people migrate to urban areas, urbanization restricts energy resources. Green investment can finance energy efficiency improvement initiatives in buildings, transportation, and other sectors. We can minimize greenhouse gas emissions and promote environmental sustainability by boosting the energy efficiency of urban areas [14]. Green investment can be crucial in financing energy-efficient initiatives, including building retrofits, public transit systems, and RE generation. Long-term economic growth requires environmental sustainability [15]:

Environmental sustainability is a multidimensional concept incorporating myriad aspects contributing to the environment’s long-term viability. The following factors determine environmental sustainability: Economic growth is commonly believed to be a primary predictor of environmental sustainability. Yet, research indicates that economic expansion can lead to environmental degradation if not adequately managed. For example, Lu [16] discovered that the evolution of the sixteen Asian economies was connected with a rise in greenhouse gas emissions. Population increase: Population growth can increase demand for natural resources and land use, which can have detrimental environmental effects. According to Research by Lambin and Meyfroidt [17], population increase was a significant factor in Amazon deforestation. Depleting natural resources such as water, forests, and minerals can have long-term detrimental environmental effects. Following a study by Acharyya [18], the overexploitation of South Asia, China, and Africa’s water resources led to the depletion of aquifers and harmful effects on ecosystems. The advancement of technology can either promote environmental sustainability or result in environmental deterioration. Nyborg, Anderies [19], further evidence is available in Wang and Shen [20] and Soga and Gaston [21].

The present study considered green investment, energy efficiency and urbanization in the equation of environmental sustainability. As our planet faces the dire consequences of environmental degradation, it has become increasingly evident that we must take immediate action. Investing in green initiatives is essential for creating a sustainable future and offers an opportunity for financial gain. It is vital to invest in green technology to halt the devastation of the environment. The world’s ever-increasing dependence on manufactured commodities has put tremendous pressure on its water, energy, and land resources. Green investments aid in restoring and preserving these vital resources, guaranteeing that the Earth will sustain life for generations [22–26]. Green investment is one of the most effective tools for reducing environmental damage. Suppose we invest in sustainable infrastructure, conservation initiatives, and alternative energy. In that case, we may be able to halt or even reverse the damage to our planet. Both the environment and the economy benefit from eco-friendly investments. Sustainable development contributes to the preservation of our natural resources, the creation of new job possibilities, and the improvement of current livelihoods. Everyone benefits. There is a complex interplay between energy efficiency and environmental damage. One positive outcome of efforts to increase energy efficiency is a decrease in the release of harmful gases. Yet, it may also cause more garbage and a rise in the use of scarce resources. Many variables affect the overall impact of energy efficiency on the environment. These include the fuel type, the technology utilized, the final use of the energy, and the method through which efficiency improvements are obtained. Reduced carbon dioxide (a greenhouse gas) emissions from power generation using less coal, for instance, might have unintended consequences for environmental quality due to increased mining and transportation. Similarly, increasing the efficiency of automobiles and trucks may save fuel and lower emissions of gases that contribute to global warming. Yet, if individuals drive more miles, the environmental benefits of this change may be nullified [27–30].

The research contributes to the existing literature in various domains. First, The Research contributes novel empirical insights into the interconnections among energy efficiency, green investment, urbanization, and environmental quality in the MENA region. This region is characterized by unique socioeconomic and environmental dynamics, and previous research focused on this specific context has been limited in scope. The work addresses a notable gap in the existing literature by analyzing the connections in the MENA area. This contribution enhances our understanding of sustainable development in this region, resulting in a more comprehensive body of knowledge. Second, the study examines the concurrent association among energy efficiency, green investment, urbanization, and environmental quality. Although previous research has examined certain aspects individually, conducting a comprehensive study that considers the interconnections among all these variables is imperative. The research provides a comprehensive perspective on the linkages. It elucidates their collective impact on environmental quality by considering multiple aspects. Third, the study’s scientific value is evident in its policy implications. The research offers valuable insights into policy choices and strategies for sustainable development in the MENA area. It achieves this by thoroughly examining the interconnections among energy efficiency, green investment, urbanization, and environmental quality. The outcomes of this study may provide valuable insights for policymakers as they seek to identify the optimal strategies for improving environmental quality while simultaneously considering factors such as energy efficiency, green investment, and urbanization. Fourthly, while the research primarily concentrates on the MENA region, it is worth noting that the outcomes and methodologies employed have implications that transcend this specific context’s confines. The study enhances the rigor and robustness of the analysis by employing various econometric methodologies, thereby expanding the analytical toolkit in sustainable development research. This research advances tools for exploring complex linkages, such as energy efficiency, green investment, urbanization, and environmental quality [31].

The motivation of the study is to gauge the effects of green investment, energy efficiency, and urbanization on environmental sustainability in MENA nations for the period 2004–2019. The key snap of the study findings is as follows. The empirical model estimation with CS-ARDL revealed contributory effects of GI, EE, and UR on ES in the long and short run. The asymmetric assessment unveiled a nonlinear linkage between explained and explanatory variables in the long and short run. The asymmetric coefficients of GI, EE, and UR revealed negative statistical significance at a 1% level, explaining the contributory role of GI, EE, and UR in environmental sustainability. Considering the study findings, policy suggestions have been formulated for further development.

The rest of the structure is as follows. The literature survey is displayed in Section II. The study’s variables’ definitions, conceptual development and methodology are available in Section IV. Empirical model estimation and interpretation reports are in Section V. Discussion is available in Section VI, and the conclusion and policy suggestion are in Section VII.

## 2. Literature survey and limitation in the existing literature

### 2.1. Green finance (investment) effects on carbon emission/ED (environmental degradation)

Similarly, heavy industries and coal-fired power plants have contributed significantly to air pollution in China. Unsustainable agricultural methods in India have damaged the country’s soil quality. The MENAS nations must prioritize green investment and environmental protection measures to overcome these concerns. Otherwise, they risk endangering their already vulnerable habitats. Using Chinese provincial data, Chen and Chen [32] assessed the effects of green finance on carbon emissions by applying the spatial dynamic panel model. This study strongly supports the fact that the development of green finance contributes a lot to reducing carbon emissions… The development of science and technology is required to strengthen the quality of green finance Bai, Chen [33]. The mixed effect of green finance on carbon emissions was analyzed in the paper of Xiong and Sun [34]. The study of Zhao, Taghizadeh-Hesary [35] examined the effect of green growth and green finance on carbon dioxide (CO2) emissions through multiple regression and found that green growth and finance greatly reduce the greenhouse effect and carbon emissions. Additionally, Meo and Abd Karim [36] confirm that green finance is the best financial strategy for mitigating carbon dioxide (CO2) emissions. The government must strengthen green finance using fiscal funding to support green investment, credit, and securities.

An analysis of the long-term equilibrium relationship between green finance, fertilizer use, and agricultural carbon emissions was conducted in the paper of Guo, Zhao [37] in China. The result of the standardized test framework supports the fact that green finance creates a significant impact on the reduction of agricultural carbon emissions. Moreover, a unidirectional causality from green finance to carbon emissions has been found, which is also consistent with the results of other tests. The affinity between green finance development, non-fossil energy consumption, and carbon intensity was developed in China [38] by applying the VECM model. The result exposes that the development of green finance is increasing the use of non-fossil energy and reducing carbon intensity. To strengthen the consumption of non-fossil energy and lowering carbon intensity, it is advisable to implement policies regarding the development of green finance [39]. The aligned findings fond in [40–42].

The effect of green finance (along with the indicators -income per capita, corporate social responsibilities, green energy, and technical innovations) on carbon emissions in E7 countries was analyzed in the research [43]. This paper’s second-generation panel cointegration method and D-H panel causality test support that green finance significantly decreases short-term and long-term carbon emissions. In the paper of [44], the factors that increase and decrease carbon emissions were analyzed based on China by applying regression. The results show that green finance development is a crucial factor that pushes carbon emissions to decline. The government should encourage green financing projects for sustainable economic growth in developing countries [45]. Analyzed the effects of green finance instruments in reducing carbon emissions in China by applying a regression model. The results reveal that green finance development (considering green credit and venture capital) significantly reduces carbon emissions. As it has been found that green credit has a strong impact on reducing carbon emissions, commercial banks should expand the green credit business.

The impact of green technology innovation and green investment on carbon emissions have been analyzed in the research of [46] based on G7 countries. The result of the cross-sectional augmented ARDL model confirms that green financing and technology innovation play significant roles in mitigating carbon emissions. It has been suggested that implementing green financing and green technology policies is crucial for the sustainable development of the countries. A similar line of findings is available in the study of [47–51]. The evaluation of the relationship between green investments, clean energy consumption, carbon emissions and economic growth was presented in the paper [52] in China. According to the result of the simultaneous equation model, it has been found that green investment affects carbon emissions to reduce, but the effect is insignificant. [53] examined the relationship between green finance and carbon emissions in China by applying the FGLS model. The result strongly supports that green finance is crucial in reducing carbon emissions; a significant negative relationship has been found. Overall, green finance development is required for the country’s sustainable economic growth.

### 2.2. Energy efficiency and environmental sustainability

There is a growing awareness of the need for energy efficiency and environmental sustainability in our society. As our population and economy continue to grow, the demand for energy increases. This places a strain on our natural resources, which can lead to environmental damage. Fortunately, many ways exist to increase energy efficiency and reduce environmental impact. We can make a big difference by making small changes in our daily lives. For example, using energy-efficient appliances, insulating our homes, and driving less can all help save energy and reduce emissions. These changes will require effort and commitment from individuals, businesses, and governments. But the benefits are clear: a healthier planet and a more sustainable future.

in the study of Akram, Majeed [54] investigated the impact of energy efficiency, RE and other factors on carbon emissions in BRICS countries by applying the nonlinear panel autoregressive distributive lag (NPARDL) model. The results confirm that energy efficiency and RE significantly reduce carbon emissions in the long run. Improvement of energy efficiency, implementation of a green growth strategy and ensuring the use of clean energy are required for environmental and economic growth. The effects of energy efficiency and utilization of RE were analyzed in the Research [55] based on G20 countries. According to the result of the fixed effect model, it has been found that, though both energy efficiency and RE create a negative impact on carbon emissions, the effect of RE on carbon emissions is greater than energy efficiency. A similar domain of literature has been posted by [56] for OECD, [57] for BRIC, and. [58] in a panel of 109 countries estimation.

In China, a study [59] analyzed the relationship between total renewable electricity generation, total hydroelectric generation, and carbon dioxide emissions. The result of the ARDL model supports that renewable electricity and hydroelectric generation significantly mitigate carbon emissions in the short and long run. The relationship between RE consumption, technological innovation, economic growth and carbon emissions was analyzed based on Denmark, Finland, Sweden, and Norway using the VAR model and Granger non-causality test [60]. The study results expose that RE consumption plays a significant role in reducing carbon emissions. In addition, a unidirectional causality from RE to carbon emissions has been found for Denmark and Finland. Conversely, a bi-directional causality between these variables has been found for Sweden and Norway. For environmental well-being, it is obvious to promote renewable energy [61]. In both the long and short run, an increase in energy efficiency pushes carbon emissions to decline. A decrease in energy efficiency increases carbon emissions. It is advisable to stimulate RE use to ensure sustainable environmental growth in developing countries. Additionaly [62], found. A positive correlation exists between non-RE consumption and carbon emissions. Besides, it has also been exposed that RE consumption has insignificant negative effects on carbon emissions, which pushes them to decline. Moreover, no significant causality exists between RE consumption and carbon emissions. However, unidirectional causality between non-RE consumption and carbon emissions has been found.

### 2.3. Urbanization and carbon emission /ED

The impact of urbanization on carbon emission efficiency was analyzed based on China in the paper [63] by applying the SFA model. The results confirm that improving the urbanization level tends to increase carbon emission efficiency, significantly reducing carbon emissions. However, excessive urbanization has also been found to increase carbon emissions by destroying the construction of a green economy [64]. The U-Kaya Identity method was applied to forecast urbanization’s effect on carbon emissions in 2020. The model results reveal that carbon emissions will increase due to the high urbanization rate. It has been suggested that industrial restructuring, technological advancement, upgrading, and implementing key energy-saving projects are crucial for ensuring a low-carbon economy [65]. The relationship between urbanization and carbon emission in West African countries was analyzed by applying Driscoll–Kraay standard errors regression and the Dumitrescu–Hurlin panel causality test. The results strongly confirm that urbanization positively impacts carbon emissions, which means carbon emissions increase due to the increased level of urbanization. Moreover, a bi-directional causality has been found between urbanization and carbon emissions. For West African countries, it is suggested to ensure technological advancement and energy efficiency to achieve sustainable economic growth.

The nexus between RE consumption, urbanization, economic growth, and carbon emissions in the Middle Eastern and North African countries was identified in the paper [66] by applying a Continuously updated, fully modified and Continuously updated bias-corrected method. The results indicate that rapid urbanization increases the level of carbon emissions, which means a positive impact of urbanization has been found on carbon emissions. As energy consumption significantly reduces carbon emissions in MENA countries, investments in green energy projects should be encouraged [67]. Zhang, Liu [68] examined the effect of economic growth, industrial structure and urbanization on carbon emission intensity in China by applying the ARDL model. The results exposed that rapid urbanization pushes the carbon emission intensity to grow, which means a positive impact has been found. In addition, a unidirectional causality has been found to exist from urbanization to carbon emissions. A similar line of evidence is available in the study of [69–71]. For the USA, [72] using the QARDL method has supported that a higher level of urbanization tends to increase carbon emissions in both the short and long run. Based on the findings, it has been suggested that controlling the detrimental effect of extreme urbanization and high natural resource rent is necessary to ensure sustainable economic growth.

Another line of evidence dealing with the nexus between urbanization and environmental sustainability is the beneficial effects of urbanization on environmental sustainability. The impacts of urbanization on carbon emissions in both the short run and long run based on OECD countries were analyzed in the paper [73]. The results of the ARDL test expose that an increased rate of urbanization pushes carbon emissions to decline. However, the impact is not that much significant. Sustainable economic and social development must promote urbanization through technological progress, optimizing energy consumption and reducing carbon emissions [74]. Examined the effects of urbanization on carbon emissions efficiency from different aspects in China by applying the IPCE model. The results support that, for mature urban agglomerations, urbanization’s population and economic and industrial effects promote carbon emission efficiency, which decreases carbon emission. However, the space expansion effect of urbanization reduces carbon efficiency. Environmental awareness should be strengthened along with urbanization to ensure a low-carbon economy. A significant negative effect of urbanization on Singapore’s carbon emissions was found in the paper [75] through the application of ARDL methodology. It does not cause environmental degradation. It is advisable for Singapore that economic growth should be prioritized rather than considering urbanization. In China [76], the contribution of Energy Service companies in reducing carbon emissions was analyzed. A relationship between urbanization, industrialization and carbon emissions was also investigated further by applying a regression model. The results say that urbanization negatively impacts carbon emissions, which means carbon emissions tend to decline due to the increasing level of urbanization. Energy-saving technology innovations are encouraged to ensure a low carbon-based economy.

## 3. Theoretical development and empirical model justification

Previous research on energy efficiency has emphasized its significance in reducing energy consumption and mitigating greenhouse gas emissions. In a study conducted by [77], the study found that advancements in energy efficiency positively impacted environmental quality within the MENA region [78]. Underscored the significance of energy efficiency in reducing pollution and mitigating the impacts of climate change. Green investment, which promotes the utilization of RE sources and sustainable technology, has been recognized as a crucial factor in achieving and maintaining environmental quality. In their study, [79] made a significant finding regarding the positive influence of green investment on environmental sustainability within the MENA region [80]. Emphasized the significance of green investment in reducing carbon emissions and fostering sustainable development. Although urbanization has been associated with economic advancement, it has also been recognized as a potential threat to environmental integrity. The utilization of energy, the emission of pollutants, and the ecological ramifications are frequently heightened within urban environments. Literature [81–83] have emphasized the importance of addressing the environmental implications of urbanization by implementing sustainable urban design, green infrastructure, and efficient resource management. [84] seeks to address and resolve potential econometric challenges during the analysis. This methodology ensures robustness in capturing the intricate dynamics and interdependencies among the factors above. Consequently, it contributes to the existing body of research and influences policy decisions about sustainable development in the MENA region [85].

## 4. Data and methodology of the study

### 4.1. Model specification and conceptual development

The motivation of the study is to assess the role of green investment, energy efficiency and urbanization for environmental sustainability in MENA notation for the period 2004–2019. It is mentioned here that the selection of panels and duration of the data purely rely on the data availability. Since the study considered balanced panel data. Therefore, we have put extra caution in data and country selection.

The targeted nexus can be displayed in the following manner.


$${ES}_{t}\int {GI}_{t}{,EE}_{t},{UR}_{t}$$ (1)

ES, GI, EE, and UR are for environmental sustainability, green investment, energy efficiency and urbanization. After transformation with the natural log of all variables, the above equation can be developed in the following regression form to derive the elasticities of explanatory variables.


$${ES(CO2)}_{,it}=\alpha_{0}+\beta_{1}{lnGI}_{it}+\beta_{2}{lnEE}_{it}+\beta_{3}{lnUR}_{it}+\epsilon_{t}+\varepsilon_{it}$$ (2)

$${ES(EF)}_{,it}=\alpha_{0}+\beta_{1}{lnGI}_{it}+\beta_{2}{lnEE}_{it}+\beta_{3}{lnUR}_{it}+\epsilon_{t}+\varepsilon_{it}$$ (3)

CO2, EF, GI, EE, and UR stand for carbon emission, ecological footprint, green investment, energy efficiency, and urbanization, respectively. The coefficients of *β*_1_, *β*_2_, *and β*_3_ explained the elasticities of explanatory variables on environmental sustainability. Table 1 displays the proxies and variables definition of the study.

**Table 1:** Proxy and variables definition.

Variables	Notation	Definition	Source
Environmental sustainability	CO2	Metric tons per capita	WDI
	Ecological footprint	gha per person	[86]
**Explanatory variables**			
Green investment	GI	Measure by investment on the environmental protection products by resident units,	OECD Statistics [87]
Energy efficiency	EE	Renewable energy sources in the total energy mix	WDI
Urbanization	UR	Measure people living in urban areas	WDI

### 4.2. Conceptual and theoretical development

Taking into account the regression equation displayed in Eq (2) and Eq (4), It is anticipated that a positive nexus will be available between green investment and environmental sustainability in MENA, suggesting that persistent green investment will prompt environmental quality by lowering the present state of carbon emission and ecological balanced that is the coefficient of GI on EE should be negative in sign. Alternatively, 1<, $\frac{ln{ES}_{,it}}{\gamma_{1}{lnGI}_{it}}$. Of the many tools at our disposal to halt the ecological decline, green investment is among the most potent. Sustainable infrastructure, conservation measures, and alternative energy can potentially reduce or even reverse the damage done to our globe. When money is put into environmentally friendly projects, it benefits the economy and the planet [88]. Natural resources are preserved thanks to sustainable development, which creates new jobs and improves current ones. So, it is a win-win situation for all parties involved. Investment in environmentally friendly technology is crucial to halt further damage to the planet. Regarding energy efficiency, the role in the environmental protection process is anticipated to be positively associated, suggesting that efficient energy sources mixed with total energy will foster the sustainability issue in environmental protection. It is projected that the coefficient energy efficiency to be negative in sign, that is, 1<, $\frac{ln{ES}_{,it}}{\gamma_{1}{lnEE}_{it}}$. Literature suggests that Climate change is frequently discussed concerning the impact of RE on carbon emissions and ecological footprint. Some argue that RE is a greener and more sustainable alternative to traditional fossil fuels. In contrast, others contend that renewables are less effective at reducing greenhouse gas emissions. A substantial corpus of scientific evidence indicates that RE can help reduce carbon emissions and ecological footprint [89, 90]. According to a study by the National RE Laboratory, wind and solar PV installations in the United States led to a net reduction of nearly 122 million metric tons of carbon dioxide equivalent (CO2e) in 2016, which is equivalent to removing more than 26 million vehicles from the road for an entire year. The study found that if all RE sources were utilized, the net CO2e reduction would be even greater [91].

As a result of no longer needing to mine or excavate for fossil fuels, the study found that land use would be drastically reduced if we switched to renewable energy. These water and land consumption reductions would substantially affect our ecological imprint [92]. The study antiquated that urbanization has a detrimental role in achieving environmental sustainability. That is, urbanization will amplify the carbon intensity and ecological imbalance. That is, the coefficient of urbanization has to be positive in sign, alternatively. $\frac{ln{ES}_{,it}}{\gamma_{1}{UR}_{it}}>1$. Literature postulated that how we plan and build our cities has a major impact on our carbon footprint and other environmental impacts. The increasing urban population strains the city’s services and facilities.

### 4.3. Estimation strategies

#### 4.3.1. Cross-sectional dependency and Homogeny test

A cross-sectional dependency test is a statistical test used to assess the relationships between variables in a data set. The test is typically used when there is no clear theoretical reason to expect a relationship between the variables. However, it is suspected that such a relationship may exist. The test can be used to examine both linear and non-linear relationships. Following the established guidelines, the present study has implemented a CSD test following the framework offered by [93, 94].

Based on the following equation, we can construct LM test statistics:

$$y_{it}=\alpha_{i}+\beta_{i}x_{it}+u_{it}\;i=1\ldots \ldots N,t=1\ldots \ldots T$$ (4)

$$LM=T\sum_{i=1}^{N-1}\sum_{j=i+1}^{N}{\hat{\rho }}_{IJ\underset{d}{\to }X^{2}N(N+1)2}$$ (5)

$${CD}_{lm}=\sqrt{\frac{N}{N(N-1)}}\sum_{I=1}^{N-1}\sum_{J=i+1}^{N}\left(T{\hat{\rho }}_{ij}-1\right)$$ (6)

$${CD}_{lm}=\sqrt{\frac{2T}{N(N-1)}}\sum_{I=1}^{N-1}\sum_{J=i+1}^{N}\left({\hat{\rho }}_{ij}\right)$$ (7)

$${CD}_{lm}=\sqrt{\frac{2}{N(N-1)}}\sum_{I=1}^{N-1}\sum_{J=i+1}^{N}(\frac{(T-K){\hat{\rho }}_{ij}^{2}-u_{Tij}}{\upsilon_{Tij}^{2}})\vec{d}(N,0)$$ (8)

Where k refers to the number of regresses, *u*_*Tij*_ and $\upsilon_{Tij}^{2}$ specifies the mean and variance of $(T-K){\hat{\rho }}_{ij}^{2}$, respectively.

Unit root test

Cross-sectionally Augmented ADF (CADF) and Cross-Sectionally Augmented IPS (CIPS) panel unit root tests are two popular methods used to test for unit roots in panel data. Both methods augment the standard ADF or IPS test by adding additional lags of the cross-sectional unit root variable, allowing for a more powerful test. The CADF test uses an augmented Dickey-Fuller regression, adding lags of the cross-sectional unit root variable until all lags are insignificant.

This approach is known as CADF. Pesaran (2007) uses Eq 9 for the CADF unit root test:

$${\Delta Y}_{it}=\beta_{i}+\gamma_{i}y_{i,t-1}+\pi_{i}{\bar{y}}_{t-1}+\beta_{i}{\bar{y}}_{t}+\rho_{it}$$ (9)

$${\Delta Y}_{it}=\mu_{i}+\gamma_{i}y_{i,t-1}+\pi_{i}{\bar{y}}_{t-1}+\sum_{k=1}^{p}\beta_{ik}{\Delta y}_{i,k-1}+\sum_{k=0}^{p}\beta_{ik}{\bar{\Delta y}}_{i,k-0}+\alpha_{it}$$ (10)

$$CIPS=N^{-1}\sum_{i-1}^{N}\partial_{i}(N,T)$$ (11)

$$CIPS=N^{-1}\sum_{i-1}^{N}CADF$$ (12)

For the Cointegration test following the error correction-based panel cointegration test, the test statistics for group statistics, i.e., *G*_*T*_ & *G*_*α*_ and panel statistics, i.e., *P*_*T*_ & *P*_*α*_, which can be extracted by executing the following equation.


$$G_{T}=\frac{1}{N}\sum_{i-1}^{N}\frac{\zeta_{i}}{SE\zeta_{i}};\;G_{a}=\frac{1}{N}\sum_{i-1}^{N}\frac{{T\zeta }_{i}}{\zeta_{i}(1)}$$ (13)

$$P_{T}=\frac{\zeta_{i}}{SE\zeta_{i}};\;P_{a}={T\zeta }_{i}$$

The generalized form of CS-ARDL takes into account the explained and explanatory variables as follows:

$$ln{ED}_{CO2,it}=\alpha_{0}+\sum_{j=1}^{q1j}\gamma_{ij}ln{ED}_{CO2,i(t-j)}+\sum_{j=0}^{q}\gamma_{1j}{lnGI}_{i(t-j)}+\sum_{j=0}^{q}\gamma_{2j}{lnEE}_{it-j}+\sum_{j=0}^{q}\gamma_{3j}{lnUR}_{it-j}+\sum_{j=1}^{q1j}\theta_{1j}ln{\bar{ED}}_{CO2,i(t-j)}+\sum_{j=0}^{q}\theta_{1j}{\bar{lnGI}}_{\left(t-j\right)}+\sum_{j=0}^{q}\theta_{2j}{\bar{lnEE}}_{t-j}+\sum_{j=0}^{q}\theta_{3j}{\bar{lnUR}}_{t-j}+\varepsilon_{it-j}$$ (14)

$$ln{ED}_{EF,it}=\alpha_{0}+\sum_{j=1}^{q1j}\gamma_{ij}ln{ED}_{EF,i(t-j)}+\sum_{j=0}^{q}\gamma_{1j}{lnGI}_{i(t-j)}+\sum_{j=0}^{q}\gamma_{2j}{lnEE}_{it-j}+\sum_{j=0}^{q}\gamma_{3j}{lnUR}_{it-j}+\sum_{j=1}^{q1j}\theta_{1j}ln{\bar{ED}}_{EF,i(t-j)}+\sum_{j=0}^{q}\theta_{1j}{\bar{lnGI}}_{\left(t-j\right)}+\sum_{j=0}^{q}\theta_{2j}{\bar{lnEE}}_{t-j}+\sum_{j=0}^{q}\theta_{3j}{\bar{lnUR}}_{t-j}+\varepsilon_{it-j}$$ (15)

Where $\bar{co2},$ $\bar{GI},\bar{EE},\bar{UR}$ exhibits the CSA of explained and explanatory variables, *α*_0_, *γ*_*ij*_ and *β*_*ij*_ explained, *θ*_1*j*_….*θ*_5*j*_; *π*_1*j*_….*π*_5*j*_ denotes the coefficients of CSA of explanatory variables on explained variables.

#### 4.3.2. Asymmetric ARDL

Following the nonlinear framework offered by Shin, Yu [95], that is, asymmetric shocks of explanatory variables [6, 96–98], the asymmetric equation for exploring the asymmetric effects of explanatory variables, which is *GI*^+^ & *GI*^−^, *EE*^+^ & *EE*^−^, *UR*^+^ & *UR*^−^

$${\Delta ED}_{CO2,it}=\beta_{0i}+\gamma_{1i}{ED}_{CO2,it-1}+\gamma_{2i}^{+}{GI}_{t-1}^{+}+\gamma_{2i}^{-}{GI}_{t-1}^{-}+\gamma_{3t}^{+}{EE}_{t-1}^{+}+\gamma_{3t}^{-}{EE}_{t-1}^{-}+\gamma_{4t}^{+}{UR}_{t-1}^{+}+\gamma_{4t}^{-}{UR}_{t-1}^{-}+\sum_{J=1}^{Q-1}\gamma_{iJ}{\Delta ED}_{CO2i,t-J}+\sum_{J=0}^{Q-1}\left(\rho_{ij}^{+}{\Delta GI}_{i,t-j}^{+}+\rho_{ij}^{-}{\Delta GI}_{i,t-j}^{-}\right)+\sum_{J=0}^{Q-1}\left(\left(\beta_{ij}^{+}{\Delta EE}_{i,t-j}^{+}+\beta_{ij}^{-}{\Delta EE}_{i,t-j}^{-}\right)\right)+\sum_{J=0}^{Q-1}\left(\xi_{ij}^{+}{\Delta UR}_{i,t-j}^{+}+\xi_{ij}^{-}{\Delta UR}_{i,t-j}^{-}\right)+\varepsilon_{it}$$ (16)

$${\Delta ED}_{EF,it}=\beta_{0i}+\gamma_{1i}{ED}_{EF,it-1}+\gamma_{2i}^{+}{GI}_{t-1}^{+}+\gamma_{2i}^{-}{GI}_{t-1}^{-}+\gamma_{3t}^{+}{EE}_{t-1}^{+}+\gamma_{3t}^{-}{EE}_{t-1}^{-}+\gamma_{4t}^{+}{UR}_{t-1}^{+}+\gamma_{4t}^{-}{UR}_{t-1}^{-}+\sum_{J=1}^{Q-1}\gamma_{iJ}{\Delta ED}_{EF,t-J}+\sum_{J=0}^{Q-1}\left(\rho_{ij}^{+}{\Delta GI}_{i,t-j}^{+}+\rho_{ij}^{-}{\Delta GI}_{i,t-j}^{-}\right)+\sum_{J=0}^{Q-1}\left(\left(\beta_{ij}^{+}{\Delta EE}_{i,t-j}^{+}+\beta_{ij}^{-}{\Delta EE}_{i,t-j}^{-}\right)\right)+\sum_{J=0}^{Q-1}\left(\xi_{ij}^{+}{\Delta UR}_{i,t-j}^{+}+\xi_{ij}^{-}{\Delta UR}_{i,t-j}^{-}\right)+\varepsilon_{it}$$ (17)

The positive and negative series can be derived by implementing the following equations.


$$\left\{ \begin{array}{c} {GI}_{i}^{+}=\sum_{X=1}^{t}{\Delta GI}_{ik}^{+}=\sum_{X=1}^{Y}MAX({\Delta GI}_{iX},0)\\ {GI}_{i}^{-}=\sum_{k=1}^{t}{\Delta GI}_{iX}^{-}=\sum_{X=1}^{T}MIN({\Delta GI}_{iX},0) \end{array}\right.;\;\left\{ \begin{array}{c} {EE}_{i}^{+}=\sum_{X=1}^{t}{\Delta EE}_{iX}^{+}=\sum_{K=1}^{Y}MAX({\Delta EE}_{iX},0)\\ {EE}_{i}^{-}=\sum_{X=1}^{t}{\Delta EE}_{iX}^{-}=\sum_{X=1}^{T}MIN({\Delta EE}_{iX},0) \end{array}\right.\;\left\{ \begin{array}{c} {UR}_{t}^{+}=\sum_{k=1}^{t}{\Delta UR}_{iX}^{+}=\sum_{X=1}^{Y}MAX({\Delta UR}_{iX},0)\\ {GG}_{t}^{-}=\sum_{X=1}^{t}{\Delta UR}_{iX}^{-}=\sum_{X=1}^{T}MIN({\Delta UR}_{iX},0) \end{array}\right.$$

## 5. Estimation and interpretation

### 5.1. Cross-sectional dependency and Homogeneity test

In this stage, we have performed a cross-sectional dependency test and slop of Homogeneity by executing the reworked instituted by. Table 2 reported the results of SHT and CSD. Inferring to the test statistics, the study established conclusive evidence by rejecting the null of cross-sectionally independence and homogeneity properties in the research units.

**Table 2:** Cross-sectional dependency and heterogeneity test.

	*LM*_*BP*_	*LM*_*PS*_	*LM*_*adj*_	*CD*_*PS*_	Δ	Adj.Δ
EF	153.039***	17.803***	128.22***	23.796***	52.095***	149.479***
CO2	348.118***	43.008***	122.913***	19.177***	62.895***	77.144***
GI	354.747***	34.776***	133.162***	19.594***	24.166***	140.143***
EE	214.29***	16.001***	108.876***	14.483***	61.466***	62.354***
UR	189.948***	27.436***	193.076***	46.472***	43.343***	117.073***

### 5.2. Panel unit root test: CADF and CIPS

The stationarity of the series is analyzed using the CADF and CIPS second-generation panel unit root tests devised by Pesaran (2007) under cross-section dependency. Panel unit root tests for the fixed and constant-trend models are summarized in Table 3. All the variables in the study are not stationary at this level. However, they are stationary at the first difference, as shown by the fixed and fixed-trend model results. All variables are verified to be integrated at the point after the first difference operation, that is, I(1).

**Table 3:** CADF and CIPS pane unit root test.

Variables	CADF		CIPS		CADF		CIPS	
	for constant		for constant		for constant and trend		for constant and trend	
	Level	1sr diff	Level	1sr diff.	Level	1sr diff.	Level	1sr diff.
EF	-2.377	-5.63***	-2.421	-3.687***	-1.673	-7.597***	-1.333	-7.779***
CO2	-1.98	-4.703***	-1.341	-4.081***	-1.212	-4.954***	-1.827	-6.289***
GI	-2.312	-6.426***	-2.743	-6.715***	-1.029	-5.178***	-1.953	-3***
EE	-1.017	-5.217***	-1.056	-4.294***	-1.278	-5.092***	-1.546	-2.531***
UR	-1.789	-2.52***	-2.501	-3.714***	-2.397	-5.915***	-2.775	-6.483***

### 5.3. Panel cointegration test

The study implemented a panel cointegration test following Westerlund [99], Kao [100], and Pedroni [101]; their results are displayed in Table 4. The study revealed that all the test statistics are statistically significant at a 1% level, suggesting rejecting the null hypothesis of no-cointegration. Alternatively, established long-run association in the empirical model.

**Table 4:** Rustles of Padroni, Kao and Westerlund cointegration test.

	ES measures by CO2			ES measures by ecological footprint		
Model	ES--->GI	ES--->EE	ES--->UR	ES--->GI	ES--->EE	ES--->UR
Gt	-11.629***	-4.732***	-10.975***	-13.824***	-10.501***	-13.43***
Ga	-11.6***	-8.215***	-9.332***	-12.615***	-9.506***	-14.09***
Pt	-12.104***	-5.95***	-10.099***	-7.412***	-13.813***	-14.839***
Pa	-14.462***	-7.454***	-12.191***	-12.627***	-13.948***	-14.351***
**KRCPT**						
MDF	-6.92***	6.248***	10.242***	11.879***	7.52***	-2.543***
DF	14.524***	9.72***	-4.285***	-7.837***	18.967***	-2.186***
ADF	-10.882***	9.992***	5.969***	-0.621***	-6.587***	-0.052***
UMDF	3.517***	-6.013***	20.524***	1.438***	-2.934***	-0.593***
UDF	-7.756***	7.627***	1.999***	12.452***	6.745***	-2.633***
**PCT**						
MDF	9.191***	2.904***	9.87***	0.694***	4.515***	0.078***
PP	-0.292***	4.432***	-2.203***	12.436***	6.734***	0.862***
ADF	12.947***	14.163***	10.89***	8.125***	11.793***	11.308***

Next, the study executed the baseline empirical model, see Table 5, through Random and Fixed effects models to initialize the effects of green investment, energy efficiency, and urbanization on environmental sustainability in MENA nations, according to the sign of coefficients of explanatory variables that GI, EE, and UR, it is apparent that GI and EE foster environmental sustainability by lowering the emission of CO2 and correcting the ecological imbalance. UR has exposed a detrimental role in establishing environmental degradation through amplifying CO2 emissions and ecological degradation.

**Table 5:** Results baseline estimation: Random effect and fixed effects.

	RE	FE	RE	FE
Model: CO2 = (GI, EE, UR)			Model: ES = (GI, EE, UR)	
GI	-0.19(0.0167)[-11.373]	-0.334(0.0262)[-12.731]	-0.394(0.0339)[11.589]	-0.072(0.0091)[7.91]
EE	-0.516(0.0563)[9.156]	-0.425(0.0644)[-6.597]	--0.325(0.0493)[-6.58]	-0.72(0.0738)[9.749]
UR	0.273(0.0519)[5.254]	-0.284(0.0241)[-11.768]	0.088(0.0067)[12.947]	0.13(0.0134)[9.673]
Constant	-1.776(0.1443)[-12.305]	-1.438(0.1629)[-8.827]	-1.296(0.1056)[-12.264]	-0.65(0.0602)[-10.796]
Control	YES	YES	YES	YES
Year	YES	YES	YES	YES
Region	YES	YES	YES	YES
R2	0.8246	0.8501	0.7921	0.8688

### 5.4. Empirical estimation: CS-ARDL

Table 6 displays the results of CS-ARDL with the proxy measures of environmental sustainability by considering carbon emission (CO2) and ecological footprint (EF).

**Table 6:** Results of cross-sectional ARDL.

	Coefficient	t-stat	std. error		Coefficient	t-stat	std. error
Model: CO2 = (GI, EE, EU, FDI, TR)				Model: EF = (GDP GDP^2^, ER, PNT, TR)			
Panel–A: Long-run Coefficients							
GI	-0.1737***	0.0095	-18.2842	GI	-0.1382***	0.0066	-20.9393
EE	-0.0748***	0.0041	-18.2439	EE	-0.0518***	0.0072	-7.1944
UR	0.0533***	0.0089	5.9887	UR	0.0359***	0.0037	9.7027
C	0.1354	0.0088	15.3863	C	0.0568	0.0094	6.0425
Panel–B: Short-run coefficients							
GI	-0.0688***	0.004	-17.2	GI	-0.0125*	0.0061	-2.0491
EE	-0.0434*	0.0112	-3.875	EE	-0.0863	0.0081	-10.6543
UR	0.0614**	0.0114	5.3859	UR	0.0799***	0.0051	15.6666
CD test		0.02272		CD test		0.02172	
Wooldridge Test for Autoco		0.968622				0.940748	
Normality test		0.970973				0.174108	
Remsey RESET test		0.78539				0.165965	

The coefficients of green investment (GI) have revealed a positive association with environmental sustainability, suggesting a negative effect following from GI to the proxy measures of ES. That is, green investment decreases the carbon intensity and establishes the ecological balance. More precisely, a 10% growth in GI will improve ES by 0.1737% through the reduction of CO2 and by 0.1382% ecological correction in the long run. Additionally, in the short run, GI amplifies ES by reducing CO2 emission by 0.688% and ecological imbalance by 0.0125%. The existing literature supports the positive tie between ES and GI, such as Zhang, Zhu [102] and Bai, Chen [33]. Guo, Zhao [37], Chen and Chen [32]. The beneficial effects of energy efficiency on environmental sustainability have been documented in the long-run and short-run assessments. Study findings suggest that the energy mix with efficient sources will improve environmental quality in the process of carbon emission reduction and ecological ramifications. In particular, a 10% change in energy mix with efficient sources that renewable sources can intensify environmental development by reducing the degradation through carbon emission by 0.748% (0.434%) and ecological destruction by 0.518% (0.863%) in the long-run (short-run) our study findings is in line with the existing literature such as [54, 55, 103–106]. The effects of RE on environmental sustainability are both positive and negative. RE sources such as solar and wind power generate electricity without air pollutants or greenhouse gas emissions. This is a major advantage over traditional fossil fuel-based power generation, which can significantly negatively impact air quality and the climate [107–113]. Additionally, RE often has a smaller footprint than traditional power generation, requiring less land and water. On the downside, RE can negatively impact the environment.

The study disclosed that urbanization fosters environmental development; that is, UR declined the rate of CO2 and ecological degradation in MENA nations. Notably, in the long run, a 10% progress in UR would increase environmental unsustainability through the induction of CO2 emission by 0.533% and ecological correction by 0.359%. Additionally, environmental degradation has been exacerbated by 0.614% and 0.799% due to CO2 emission and ecological instability in the short-run, which is supported by the study of [64, 65]; however, confronts the literature offered in the study of [73, 75, 76, 107–109].

### 5.5. Long-run and short-run coefficients of asymmetric ARDL

Next, Table 7 displays the results of the asymmetric assessment for documenting the asymmetric coefficients of GI, EE, and UR on ES. Panel-A reports the asymmetric coefficients in the long run, and Panel–B for the short-our coefficient.

**Table 7:** Results of asymmetric coefficients.

Variables	Coefficient	std. error	t-stat	Coefficient	std. error	t-stat
Model: CO2 = (GI+, GI-, EE+, EE-, EU+, EU-)				Model: EF = (GI+, GI-, EE+, EE-, EU+, EU-)		
Panel–A: long-run asymmetric coefficients						
GI⁺	-0.0718	0.0272	2.63971	-0.0856	0.0615	-1.3918
GI	-0.0755	0.0456	1.6557	-0.076	0.0463	-1.6414
EE⁺	-0.1408	0.0788	1.7868	-0.0976	0.0631	-1.5467
EE־	-0.1417	0.047	3.01489	-0.0896	0.0657	-1.3637
UR⁺	0.0857	0.0853	1.00469	0.0906	0.0468	1.9358
UR־	0.1161	0.0649	1.78891	0.0682	0.0574	1.1881
C	0.1402	0.0466	3.00858	0.0837	0.0841	0.9952
Panel–B: Short-run coefficient						
GI⁺	-0.0251	0.0079	-3.17722	-0.0355	0.00451	-7.8713
GI	-0.0389	0.0032	-12.0433	0.0017	0.0028	0.6071
EE⁺	-0.0021	0.0061	0.3471	-0.0194	0.00689	-2.8156
EE־	-0.0051	0.0053	0.9604	-0.014	0.00718	-1.9498
UR⁺	0.0131	0.0054	2.4169	-0.0088	0.00447	-1.9686
UR־	0.0106	0.0025	4.0926	-0.0062	0.00496	-1.2501
cointEq (-1)	-0.4306	0.00819	-52.5763	-0.4021	0.0829	-4.85042

Referring to asymmetric coefficients of green investment (GI^+^ & GI^-^), the positive (negative) shocks of GI revealed negative and statistically significant in the long run with a coefficient of -0.0718(-0.0755) and short-run with a coefficient of -0.0251(-0.0389) where CO2 considered as a measure of ES. Furthermore, in the case of ES measured by ecological footprint, the study exposed the asymmetric shock of GI established adversely associated with a coefficient of -0.0856(0.0761) in the long run and with a coefficient of -0.0355 in the short-run, be noted that adverse shocks have found statistically insignificant. Considering the asymmetric findings, the study advocated that mobilizing and channeling the investment in environmental protection will have a greater impact on environmental development in the long and short run. The asymmetric assessments revealed a negative and statistically significant linkage between asymmetric shocks in EE and ES, measured by CO2 and ecological footprint. In particular, a 10% positive (negative) shock, in the long run, resulted in the acceleration of environmental sustainability by reduction of carbon emission by 1.408%(1.417%) and improvement in the ecological correction by 0.976%(0.896%). For the short-run case, the asymmetric shocks of EE revealed a statistically insignificant tie to carbon emission. In contrast, the statistically significant association revealed to ecological footprint is that ecological stability has improved (declined) at a rate of 0.194%(0.014%) with a 10% change in energy efficiency. Urbanization has destructive effects on environmental sustainability. The asymmetric shock in UR disclosed positive statistically significant in the long-run(short-run) evaluation. Precisely, a 10% positive(negative) variation in UR established further degradation (improvement) in environmental quality by 0.875%(1.161%) through the concentration of CO2 in the environment and by 0.906% (0.682%) through ecological ramification. For the short-run, asymmetric shocks of UR are positively connected to CO2 and negatively associated with the ecological footprint [114–117].

The results of the standard Wald test for assessment of long-run and short-run asymmetry are displayed in Table 8 with the null of symmetry. The study disclosed that all the test statistics were statistically significant, confirming the null rejection. Alternatively, established asymmetric relations between explanatory variables with environmental sustainability.

**Table 8:** Results of long-run and short-run asymmetry test.

	ES measures by Co2		ES measures by Ecological footprint	
Wald test	Test statistics	Remarks	Test statistics	Remarks
$W_{LR}^{GI}$	5.478		6.802	
$W_{SR}^{GI}$	11.956		7.61	
$W_{LR}^{EE}$	9.156		9.007	
$W_{SR}^{EE}$	4.297		2.547	
$W_{LR}^{UR}$	9.837		11.144	
$W_{SR}^{UR}$	11.155		13.523	

The study has implemented AMG, CCE, and MG regression to test the robustness, especially for explanatory variables on ES. The results of the robustness test are displayed in Table 9. The study confirmed empirical robustness by supporting the earlier model estimation by referring to the GI, EE, and UR signs.

**Table 9:** Robustness test: AGM, CCE, MG.

	AGM	CCE	MG
Model: CO2 = (GDP GDP2, ER, PNT, TR)			
GI	-0.0657(0.008)[-7.465]	-0.0645(0.004)[-16.125]	-0.1066(0.003)[-27.333]
EE	-0.0588(0.006)[-9.333]	-0.1162(0.011)[-9.931]	-0.0289(0.008)[-3.481]
UR	0.0589(0.009)[6.402]	0.0441(0.003)[14.7]	0.1453(0.008)[16.325]
C	0.0207(0.008)[2.406]	0.0204(0.004)[4.163]	0.0922(0.004)[21.441]
Wald test	0.0068	0.0047	0.0084
CD test	0.0021	0.0108	0.0046
Model: ES = (GDP GDP^2^, ER, PNT, TR)			
GI	-0.0356(0.011)[-3.095]	-0.0548(0.008)[-6.447]	-0.1406(0.005)[-28.12]
EE	-0.0292(0.006)[-4.562]	-0.0973(0.002)[-42.304]	-0.1793(0.01)[-17.24]
UR	0.0447(0.01)[4.257]	0.0916(0.01)[8.98]	0.1483(0.008)[17.447]
C	0.0357(0.008)[4.011]	0.0906(0.003)[25.885]	0.1551(0.006)[23.149]
Wald test	0.0091	0.0119	0.0058
CD test	0.0119	0.0119	0.0024

## 6. Discussion of the findings

The coefficients of green investment in MENA have been established as positively connected to environmental sustainability, suggesting the beneficial effects of managing environmental adversity through green investment, supported by [34, 42, 118]. The effects of green investment on carbon emissions are both significant and far-reaching. In terms of reducing emissions, green investment is one of the most important things we can do. Not only does it help to reduce the number of greenhouse gases in the atmosphere, but it also helps to create jobs and economic growth. In terms of its effect on climate change, green investment is vital. It helps reduce the amount of carbon dioxide and other greenhouse gases in the atmosphere, contributing to global warming [119, 120]. Additionally, green investment helps to create jobs and spur economic growth. This is important because a strong economy must fund further research and development to find new ways to reduce emissions [116, 121–123]. Thus, green investment is essential to combating climate change and reducing carbon emissions. We must continue to invest in it if we want to make a difference. In addition, several of these firms’ products, such as oil and gas, are responsible for significant environmental damage. For instance, oil spills may significantly damage marine life and coastal ecosystems. At the same time, gas flaring emits vast volumes of greenhouse gases into the atmosphere. Encouraging green investment to combat climate change and advance toward a more sustainable future is crucial. Yet, it is also essential to consider these expenditures’ potential adverse environmental effects. In conclusion, green investment is essential for the future of our planet by helping to reduce environmental degradation. Investing in RE sources and reducing one’s carbon footprint can help ensure that our Earth remains healthy and habitable for future generations. While there are many ways to invest in green initiatives, it is essential to research before committing funds to be sure that the money will be put towards meaningful causes that benefit both people and nature alike.

The beneficial effects of energy efficiency on environmental sustainability have been documented in the long-run and short-run assessments. Study findings suggest that the energy mix with efficient sources will improve environmental quality in the process of carbon emission reduction and ecological ramifications. In particular, a 10% change in energy mix with efficient sources that renewable sources can intensify environmental development by reducing the degradation of carbon emission by 0.748% (0.434%) and ecological destruction by 0.518% (0.863%) in the long-run (short-run) our study findings is in line with the existing literature such as [54, 55, 103–106]. RE is one of the most important drivers of environmental sustainability. RE is sustainable and does not deplete the earth’s resources. This means that it is a critical ingredient in the fight against climate change and in protecting our planet. There are many types of renewable energy, each with advantages and disadvantages. Solar energy is perhaps the most well-known form of renewable energy, and it has the potential to be very efficient and cost-effective [57, 119, 120, 124]. However, solar panels require much space and can be expensive to install. Wind energy is another popular form of renewable energy. However, it too has its drawbacks–wind turbines can be noisy, and they can kill birds that fly into them. Despite these challenges, RE is crucial for the future of our planet. It is clean, sustainable, and renews itself continually. We must continue to explore and invest in new technologies that will help us harness the power of renewables and make our world a cleaner, healthier place for generations to come. [61, 62].

Urbanization hurts the environment sustainably, indicating the detrimental role of environmental quality through excessive carbon emission and ecological imbalance in the ecosystem. Notably, in the long run, a 10% progress in UR would increase environmental unsustainability through the induction of CO2 emission by 0.533% and ecological correction by 0.359%. Additionally, environmental degradation has been exacerbated by 0.614% and 0.799% due to CO2 emission and ecological instability in the short-run, which is supported by the study of [64, 65]; however, confronts the literature offered in the study of [73, 75, 76]. As the world’s population continues to grow and urban areas continue to expand, it is essential to consider the impact of this growth on the environment. Urbanization can lead to increased pollution and waste and a higher demand for resources such as water and energy. If not managed properly, this can strain the local environment and lead to serious sustainability issues. Fortunately, several things can be done to help make urban areas more sustainable. For example, increasing the use of public transportation, encouraging green space and parks, and promoting energy efficiency can all help reduce the impact of urbanization on the environment. Additionally, it is essential to educate people about sustainability so that they can make informed decisions about how to live in an urban area in an environmentally responsible way [114, 122].

## 7. Conclusion and suggestions

### 7.1. Conclusion

The key findings of the study are as follows. First, the cross-sectional dependency and slope of homogeneity test results revealed that research units had shared typical dynamics and heterogeneity properties. Second, the stationary test following CIPS and CADF exposed all the variables to be stationary after the first difference. Third, the panel cointegration test established a long-run association between GI, EE, UR, and ES in MENA nations. Fourth, the empirical model estimation with CS-ARDL, the study disclosed contributory effects of GI, EE, and UR on ES both in the long run and short run. Fifth, the asymmetric assessment unveiled a nonlinear linkage between explained and explanatory variables in the long and short run. The asymmetric coefficients of GI, EE, and UR revealed negative statistical significance at a 1% level, explaining the contributory role of GI, EE, and UR in environmental sustainability.

### 7.2. Policy suggestions

First, there are many ways to improve environmental sustainability through green investment in MENA. One way is to invest in RE sources such as solar and wind power. Another way is to invest in green infrastructure projects such as energy-efficient buildings and public transportation systems. Additionally, green investment can fund research and development of new clean technologies. One of the most important things individuals can do to support environmental sustainability is to invest in green companies and products. Doing so, you help support the growth of environmentally friendly businesses and encourage other companies to adopt more sustainable practices. There are many ways to make green investments, including through traditional financial channels such as stocks and bonds or impact investing platforms that specifically target companies with a positive environmental impact. No matter how you choose to invest, it is important to research to ensure that your money goes towards companies and projects committed to making a difference for the environment. With suitable green investments, we can all play a part in creating a more sustainable future for our planet.

Furthermore, there exists a multitude of strategies that can be employed to enhance environmental sustainability by optimizing energy efficiency. One effective strategy entails the utilization of energy-efficient appliances and lighting solutions. An alternative method involves implementing insulation measures within residential or commercial structures, aiming to mitigate heat loss during winter months and minimize heat gain during summer periods. In addition to implementing energy-saving measures such as sealing air leaks and utilizing a programmable thermostat, one can effectively conserve energy. Another strategy for enhancing environmental sustainability involves utilizing RE sources, specifically solar or wind power. Solar panels can harness solar energy and convert it into electricity, thereby offering a sustainable and renewable power source. On the other hand, solar water heaters utilize solar energy to heat water, eliminating the need for traditional fossil fuel-based heating methods. In addition to their primary function, wind turbines can harness the kinetic energy of wind and convert it into electrical energy. One can effectively mitigate their environmental footprint by adopting a reduced frequency of vehicular travel. Carpooling, walking, and biking are highly commendable modes of transportation that effectively mitigate gasoline consumption. One effective strategy to reduce transportation expenses is to opt for accommodation close to one’s workplace or educational institution. In order to enhance environmental sustainability, it is imperative to adopt the practice of recycling and composting materials as opposed to their disposal in landfills. Recycling serves to mitigate the demand for fresh materials, thereby contributing to resource conservation. Simultaneously, composting plays a crucial role in curbing the release of greenhouse gas emissions from the decomposition of organic matter.

Furthermore, with the ongoing global urbanization process, it is imperative to thoroughly contemplate the environmental sustainability of urban areas. As the population in urban areas continues to grow, there is an increasing demand for resources and services, thereby exerting additional pressure on the environment. Various strategies can be implemented to enhance the sustainability of cities. These include the promotion of green spaces, the utilization of RE sources, and the enhancement of waste management systems. Urbanization can potentially result in various detrimental impacts on the environment, including but not limited to air pollution, water pollution, and noise pollution. It is imperative to undertake measures to mitigate these impacts to enhance the sustainability of urban areas. One potential approach to address this issue is promoting green spaces within urban areas. This can offer numerous advantages, including reducing air pollution and providing habitat for wildlife. Another method for enhancing environmental sustainability involves the utilization of RE sources. This has the potential to effectively mitigate emissions from power plants and other significant sources of pollution. Finally, the enhancement of waste management practices can contribute to promoting urban sustainability. By diverting waste from landfills and incinerators, it is possible to effectively mitigate the emission of greenhouse gases into the atmosphere. Numerous measures can be implemented to enhance the environmental sustainability of cities. By advocating for the expansion of green spaces, the utilization of RE sources, and the enhancement of waste management protocols, we have the potential to profoundly influence the sustainability of our urban environments.
